# Effect and Related Mechanism of Platelet-Rich Plasma on the Osteogenic Differentiation of Human Adipose-Derived Stem Cells

**DOI:** 10.1155/2022/1256002

**Published:** 2022-08-08

**Authors:** Jufang Chen, Yuanyuan Zhang, Mingjin Liu, Zongyuan Zhou, Qianwen Li, Tianjiao Huang, Yang Yue, Yulou Tian

**Affiliations:** Department of Orthodontics, School and Hospital of Stomatology, China Medical University, Liaoning Provincial Key Laboratory of Oral Diseases, No. 117 Nanjing North Street, Heping District, Shenyang, 110000 Liaoning Province, China

## Abstract

**Objective:**

Human adipose-derived stem cells (hADSCs) are ideal seed cells for the regeneration of alveolar bone defects. Platelet-rich plasma (PRP), which is rich in growth factors, promotes tissue repair. The purpose of the present study was to investigate whether PRP promotes the osteogenic differentiation of hADSCs and to perform high-throughput sequencing to explore the possible mechanism.

**Methods:**

hADSCs were divided into the three following groups: CON group, OM group, and PRP group. Osteogenesis was detected by Alizarin Red staining on day 14. Total RNA was extracted from the OM and PRP groups for high-throughput sequencing. The target genes of the differentially expressed osteogenic-related miRNAs were predicted, and combined miRNA/mRNA analysis was then performed. The mRNA and protein expression levels of hsa-miR-212-5p, type 1 cannabinoid receptor (CNR1), alkaline phosphatase (ALP), Runx2, osteocalcin (OCN), and collagen 1 A1 (COL1A1) in the OM and PRP groups were detected by qRT–PCR and Western blot analyses. The binding between hsa-miR-212-5p and CNR1 was detected by a dual-luciferase reporter assay.

**Results:**

Both the OM and PRP groups exhibited enhanced proliferation of hADSCs, and the differences at 48 h and 72 h were statistically significant (*P* < 0.05). The PRP group had significantly more calcium nodules than the CON group (*P* < 0.05). Through high-throughput sequencing analysis, differential miRNA and mRNA expression profiles were obtained. During hADSC osteogenesis, the expression of hsa-miR-212-5p was downregulated, and the expression of CNR1 was upregulated. hsa-miR-212-5p was found to bind directly to the 3′ UTR of CNR1.

**Conclusions:**

The present findings indicated that downregulation of hsa-miR-212-5p and upregulation of CNR1 may be involved in the process by which PRP promotes the osteogenic differentiation of hADSCs.

## 1. Introduction

Alveolar bone defects mainly manifest as thin alveolar bone plates, “bone windows,” and “bone cracking,” which have a high prevalence in all types of malocclusion patients [1]. Alveolar bone defects may be further exacerbated with orthodontic treatment, which not only limits the movement range of teeth but also affects health and beauty, which are some of the major challenges for orthodontists. At present, guided bone regeneration, periodontal accelerated osteogenic orthodontics, and other methods are often used in the clinical treatment of alveolar bone defects. Conventional surgery for alveolar bone defects is traumatic [2] and may be a poor strategy in terms of long-term stability [3]. Bone tissue engineering technology has proposed a new scheme for the treatment of alveolar bone defects, and the experimental exploration of the regeneration and repair of alveolar bone defects is of great significance for improving the effect of orthodontic treatment, expanding the range of tooth movement, and improving the comfort of patients. Bone marrow mesenchymal stem cells (BMSCs) efficiently facilitate bone regeneration [4, 5] and are the most widely studied seed cells in bone tissue engineering [6, 7]. However, the yield of the extracted stem cells is low, and the extraction process is painful.

Adipose-derived stem cells (ADSCs) can be obtained in large quantities from resected adipose-derived tissue or through liposuction with little damage to the donor site, and they are similar to BMSCs in terms of gene expression and osteogenic ability [8]. The yield and proliferation capacity of ADSCs are also higher than those of BMSCs [9, 10]. ADSCs have gradually attracted attention and have become a promising stem cell type for bone tissue engineering and an ideal seed cell type for the treatment of alveolar bone defects.

Platelet-rich plasma (PRP) is obtained by increasing the concentration of platelets in plasma by removing red blood cells [11]. In recent years, the role of PRP in bone defects has gradually attracted attention [12]. Tajima et al. [13] demonstrated that 5% PRP significantly induces ADSCs to secrete growth factors, and the combined use of ADSCs and PRP significantly promotes the repair of rat skull defects.

MicroRNAs (miRNAs) are 18- to 26 bp endogenously initiated noncoding RNAs that regulate posttranscriptional gene expression through specific base pairing between the 5′ end and the 3′ untranslated region of the target gene [14, 15], and they play important regulatory roles in organisms. For example, miR-26a-5p regulates the osteogenic differentiation of ADSCs through the Wnt5a/Ca2+ signaling pathway [16], and miR-145-5p inhibits the osteogenic differentiation of ADSCs by targeting signaling protein 3A [17]. miR-1249-5p promotes the osteogenic differentiation of ADSCs by targeting PDX1 through the PI3K/Akt signaling pathway [18]. The miR-135/HOXA2/Runx2 pathway may contribute to the regulation of osteogenic differentiation and bone formation of ADSCs, and miR-135-modified ADSC and scaffold complexes are effectively used to repair bone defects of critical size [19]. Studies have shown that a variety of miRNAs are involved in the osteogenic differentiation of ADSCs, and that the regulatory mechanism is complex. However, many miRNAs in the ADSC osteogenic regulatory gene network have not yet been discovered.

In the present study, hADSCs were induced with osteogenic differentiation medium (OM) supplemented with 5% PRP to observe the promoting effect of PRP on the osteogenesis of hADSCs and detect the expression of Runx2. The expression profile of differential miRNAs and the mRNA expression profile associated with PRP promoting hADSC osteogenesis were explored by high-volume sequencing technology, and the osteogenic genes were screened out and verified by qRT–PCR, providing a basis for further research on the mechanism of miRNAs in PRP-induced hADSC osteogenesis. The present study provides a preliminary foundation for the clinical transformation of ADSCs in the treatment of alveolar bone defects.

## 2. Materials and Methods

### 2.1. Preparation of PRP

The whole blood samples used in this study were collected from volunteers who had no infectious or systemic diseases. After obtaining the approval of the Ethics Committee of China Medical University and the informed consent of the volunteers, 400 ml of blood was collected intravenously from each volunteer. At room temperature, the whole blood was centrifuged for 10 min at 377 g, resulting in the following three layers: upper layer, which was plasma; middle layer, which was white blood cells and platelets; and lower layer, which was red blood cells. The upper and middle layers were collected. The sample was centrifuged at 1509 g for 20 min, and the bottom precipitate (PRP) was collected.

### 2.2. Identification of Stem Cell Properties

#### 2.2.1. Identification of the Immunophenotype

Third-generation hADSCs were collected and prepared into cell suspensions after cells reached 80%-90% confluence. Cells were divided into 6 flow tubes with the number of cells adjusted to 1 × 10^6^ per tube, and the tubes were divided into the control group, CD34-PE group, CD45-FITC group, CD73-PE group, CD90-PE group, and CD105-PE group. Fluorescently labeled antibodies (Biolegend, USA) were added to each group except the control group. The samples were incubated at room temperature in the dark, washed with PBS (Gibco, USA), resuspended in 500 *μ*l of PBS, and then detected by flow cytometry.

#### 2.2.2. Multilineage Assay

According to the manufacturer's instructions (Cyagen, USA), multiple differentiation capabilities were identified. To verify the osteogenesis ability, when third-generation hADSCs reached 60%-70% confluence in serum-free cell culture medium supplemented with 10% FBS, the OM was replaced every 3 days for a total of 21 days, and cells were then stained with Alizarin Red. To verify the adipogenic ability, third-generation hADSCs were cultured until 100% confluency, and the medium was replaced with adipogenic differentiation medium A. After 3 days of induction, liquid A was replaced with liquid B. After 24 h of culture, liquid B was replaced with liquid A. The culture medium was alternated between liquid A and liquid B five times. Cells were cultured for 28 days and stained with Oil Red O. To verify the chondrogenic differentiation ability of hADSCs, 3.5 × 10^5^ cells were resuspended in 0.5 ml of premixed solution of chondrogenic differentiation medium and then centrifuged at 150 g for 5 min. Cells were then added to 0.5 ml of chondroblast induction medium, resuspended, and centrifuged. The medium was changed every 3 days, and cells were cultured for 28 days. Cells were then fixed with formalin and stained with Alcian blue.

### 2.3. Cell Culture and Grouping

hADSCs were purchased from Shenyang Cell Therapy Engineering Technology Research Centre Company. Serum-free cell culture medium (Lonza, USA) supplemented with 10% foetal bovine serum (FBS; Gibco, USA) was used to culture cells at 37°C in a 5% CO_2_ incubator. In subsequent experiments, hADSCs were divided into the following three groups for culture: CON group (negative control group, which was cultured with serum-free cell culture medium supplemented with 10% FBS), OM group (positive control group, which was cultured with hADSC OM), and PRP group (experimental group, which was cultured with hADSC OM supplemented with 5% PRP).

### 2.4. Measurement of hADSC Proliferation Ability by the Cell Counting Kit-8 (CCK-8) Assay

Third-generation hADSCs were collected and seeded into 96-well plates at 4000 cells/well in 100 *μ*l of serum-free cell medium containing 10% FBS. When cells reached 60%-70% confluence, the culture medium was changed as follows: the CON group medium was replaced with serum-free cell medium containing 10% FBS, the OM group medium was replaced with adult ADSC OM, and the PRP group was replaced with adult ADSC OM containing 5% PRP. Cells were cultured for 24 h, 48 h, and 72 h. Then, 10 *μ*l of CCK-8 solution (Solarbio, Beijing) was added to each well, and the samples were incubated at 37°C for 2 h. The absorbance value A at 450 nm was measured with a microplate analyser.

### 2.5. Evaluation of hADSC Osteogenic Differentiation Ability by Alizarin Red Staining

Third-generation hADSCs were seeded in a 6-well plate at a density of 2 × 10^4^ cells/cm^2^ in 2 ml of serum-free cell medium containing 10% FBS. Cells were divided into the following groups with three replicate wells per group: CON group, OM group, and PRP group. After 14 days of induction, Alizarin Red staining was performed to detect osteogenesis. After discarding the supernatant, 10% cetylpyridinium chloride solution (Meilun Biotechnology, China) was added, and the mixture was placed at room temperature for 30 min. The absorbance was measured at 562 nm using an ultraviolet (UV) spectrophotometer. Each sample was assessed three times, and the mean and standard deviation were calculated.

### 2.6. miRNA and mRNA Sequencing

hADSCs were seeded into 10 cm petri dishes at a density of 2 × 10^4^ cells/cm^2^, and the OM and PRP groups were set up with three replicates per group. After 14 days of osteogenic induction, the culture medium was aspirated, and 1 ml of TRI Pure was added to each petri dish to extract total RNA. miRNA sequencing and mRNA sequencing were performed in a blinded manner by Hangzhou Lianchuan Biotechnology Co., Ltd.

Two software programs, TargetScan (v5.0) [20] and miRanda (v3.3a) [21], were used for target gene prediction of 43 significantly different miRNAs, and the intersection of the two software program datasets was used as the final target gene set for the differential miRNAs. The literature was searched, and the GO terms and pathway names related to osteogenesis were sorted. The genes related to osteogenesis were screened out followed by enrichment and analysis using the Lianchuan Biological Cloud Platform with cloud tools (https://www.omicstudio.cn/login).

According to the sequencing results, the differentially expressed genes, hsa-miR-204-3p, hsa-miR-212-5p, hsa-miR-495-3p_r+1, leptin (LEP), gremlin 1 (GREM1), and type 1 cannabinoid receptor (CNR1), were selected from 28 reverse regulatory relationships for qRT–PCR verification. The primer sequences are listed in Table 1.

### 2.7. qRT-PCR Detection of the Expression of hsa-miR-212-5p, CNR1, and Osteogenesis Markers

On day 14 of osteogenic induction, total RNA of the OM and PRP groups was extracted using TRI Pure lysis solution (Bioteke, China), and the RNA concentration was measured using an UV spectrophotometer (Thermo, USA). According to the instructions (Biyuntian, China), the RNA samples were reverse transcribed to obtain cDNA. Quantitative analysis was performed using an Exicycler 96 quantitative fluorescence analyser (Bioneer, Korea), and the relative expression levels were calculated using the 2^-△△CT^ method. The primer sequences are listed in Table 1.

### 2.8. Western Blot Analysis

On day 14 of osteogenic induction, lysis solution was added to the OM and PRP groups to extract protein, and protein quantification was performed using a BCA kit (Wanleibio, China). Proteins were isolated by electrophoresis using an SDS–PAGE gel kit (Wanleibio, China) and then transferred to a PVDF membrane (Millipore, USA). The membrane was blocked with 5% skimmed milk powder (Yili, China) for 1 h and then incubated with primary antibody. The following primary antibodies were used: alkaline phosphatase (ALP) (Abclonal, China), Runx2 (Wanleibio, China), OCN (Affinity, China), COL1A1 (Wanleibio, China), CNR1 (Abclonal, China), and *β*-actin (Wanleibio, China). After four washes (5 min each), the membrane was then incubated with secondary antibody. The membrane was washed six times with Western detergent (Wanleibio, China), and enhanced chemiluminescence (ECL) solution (Wanleibio, China) was applied for exposure in a dark room. The film was scanned, and the optical density of the target protein was analyzed with Gel-Pro Analyser software.

### 2.9. Dual-Luciferase Activity Assay

After reaching 90% confluence, 293 T cells (iCell Bioscience Inc., China) were washed with PBS, digested with trypsin (Sigma, USA), resuspended, cultured for 24 h, and transfected. Solution A was prepared by mixing 50 *μ*l of Opti-MEM (Invitrogen, USA) and 3 *μ*l of Lipofectamine 3000 (Invitrogen, USA). Solution B was prepared by mixing 50 *μ*l of Opti-MEM, 2 *μ*l of P3000, 15 pmol sequence, and 0.5 *μ*g of plasmid. Solution A was mixed with solution B and added dropwise to the wells. The plate was then shaken, and luciferase activity was detected 48 h after transfection using a luciferase assay kit (KaijiBio, China).

### 2.10. Statistical Analysis

SPSS Statistics 26.0 software was used for all statistical analyses. Multivariate analysis of variance was performed to evaluate the results of the CCK-8 assay, and Bonferroni correction was used in pairwise comparisons. Statistical analysis of the qRT–PCR results was conducted using a *t*-test. *P* < 0.05 indicated a statistically significant difference.

## 3. Results

### 3.1. Characterization and Identification of hADSCs

After 24 h of cell resuscitation and culture, hADSCs were observed microscopically, and the cells were reticulated or fusiform, which was consistent with the adherent growth characteristics of mesenchymal stem cells. When cultured to the third generation, hADSCs grew well with long spindle-shaped, polygonal, and swirl-shaped growth (Figures 1(a) and 1(b)). Flow cytometry results showed that the cells were positive for surface markers of mesenchymal stem cells (CD73, CD90, and CD105) and negative for surface markers of haematopoietic stem cells (CD34 and CD45) (Figure 1(c)). The experimental results for multidirectional differentiation showed that hADSCs induced osteogenic differentiation, adipogenic differentiation, and chondrogenic differentiation (Figures 1(d)–1(f)). These results indicated that the cells used in this study meet the international standards of ADSCs.

### 3.2. PRP Promotes the Proliferation of hADSCs and the Formation of Calcium Nodules

The CCK-8 results showed that compared to the CON group, both the OM and PRP groups showed enhanced proliferation ability of hADSCs, and the differences at 48 h and 72 h were statistically significant (*P* < 0.05). However, there was no statistically significant difference between the OM and PRP groups (*P* > 0.05), indicating that PRP had no cytotoxicity (Figure 2(d)). Alizarin Red staining showed that both OM and PRP induced osteogenic differentiation of hADSCs, and the PRP group had more calcium nodules, which demonstrated that PRP further promoted the osteogenic differentiation of hADSCs based on OM induction (Figures 2(a)–2(c)). qRT–PCR analysis indicated that the expression level of Runx2 in the PRP group was significantly higher than that in the OM group (*P* < 0.05) (Figure 2(e)).

### 3.3. miRNA and mRNA Sequencing Results

The miRNA sequencing results showed that a total of 816 differential miRNAs were identified between the PRP and OM groups. The expression profile of differentially expressed miRNAs is shown in Table 2, and the heat map of differentially expressed miRNAs is shown in Figure 3(a). Taking the intersection of the prediction results of TargetScan and miRanda, a total of 12,115 target genes were predicted among 43 miRNAs with significant differences (*P* < 0.05), and there were 106,766 miRNA/mRNA regulatory relationships. The results of GO enrichment analysis of differential miRNA target genes are shown in Figure 3(b). The results of mRNA sequencing showed that a total of 60,612 genes were detected in the PRP and OM groups, among which 1146 genes were significantly differentially expressed (*P* < 0.05), and a volcano map was generated for all the differentially expressed genes (Figure 3(c)). According to the GO terms, 156 genes related to osteogenesis were further screened out from 1146 differentially expressed genes, and GO enrichment analysis was conducted (Figure 3(d)). The KEGG enrichment analysis results were analyzed by GGplot2 and are presented in a scatter diagram (Figure 3(e)). Taking FPKM ≥ 10 as the limiting threshold, 20 osteogenic genes were further screened out from 156 osteogenic genes. The mRNA expression profiles of PRP promoting the osteogenic differentiation of hADSCs are shown in Table 3. According to the prediction results of miRNA target genes, 20 osteogenic genes were selected. A total of 28 reverse regulatory relationships were obtained. The regulatory relationships of miRNA/mRNA osteogenesis are shown in Table 4, and the analysis of miRNA and mRNA sequencing results and the flow chart of miRNA/mRNA combined analysis are shown in Figure 3(f).

The qRT–PCR verification results were contrary to the sequencing results. The qRT–PCR verification results showed that the expression level of hsa-miR-204-3p was downregulated (*P* < 0.05), while the sequencing results showed that the expression level of hsa-miR-204-3p was upregulated (*P* < 0.05). The qRT–PCR validation results of hsa-miR-212-5p, hsa-miR-495-3p_r+1, LEP, GREM1, and CNR1 were consistent with the sequencing results (Figure 4).

### 3.4. hsa-miR-212-5p Is Downregulated, and CNR1 Is Upregulated during Osteogenic Differentiation of hADSCs

To confirm that PRP promotes the osteogenic differentiation of hADSCs at the molecular level and to explore the mechanism of action of hsa-miR-212-5p and CNR1, we detected the expression of hsa-miR-212-5p and CNR1 in the OM and PRP groups on day 14 and detected the expression of the ALP, Runx2, OCN, and COL1A1 osteogenic markers. The qRT–PCR results showed that the expression of osteogenic markers and CNR1 was upregulated but that the expression of hsa-miR-212-5p was downregulated (Figure 5(a)). The Western blot results were consistent with the qRT–PCR results (Figure 5(b)). Therefore, we concluded that PRP promotes the osteogenic differentiation of hADSCs, and that hsa-miR-212-5p is downregulated, and CNR1 is upregulated during this process.

### 3.5. hsa-miR-212-5p Targets CNR1

We found a hsa-miR-212-5p-binding site in the 3′ UTR of CNR1 (Figure 5(c)). To assess whether hsa-miR-212-5p directly targets CNR1, a dual-luciferase assay was performed, which demonstrated that hsa-miR-212-5p mimics significantly inhibited luciferase activity in the wild-type (WT) group (*P* < 0.05) but had no significant effect on luciferase activity in the mutant (MUT) group (*P* > 0.05) (Figure 5(d)). These results suggested that hsa-miR-212-5p directly targets the 3′ UTR-specific binding sites of CNR1.

## 4. Discussion

In the present study, PRP was selected as a stimulating factor for the osteogenic differentiation of hADSCs. Alizarin Red staining and quantitative analysis showed that PRP promoted the formation of calcium nodules. qRT–PCR and Western blot analyses demonstrated that the expression of the ALP, Runx2, OCN, and COL1A1 osteogenesis markers was upregulated. Therefore, these results indicated that PRP promotes the osteogenic differentiation of hADSCs, that the expression of hsa-miR-212-5p is downregulated, and the expression of CNR1 is upregulated during this process. The dual-luciferase assay demonstrated that hsa-miR-212-5p bound to the 3′ UTR-specific site of CNR1. Thus, these findings suggested that the downregulation of hsa-miR-212-5p and the upregulation of CNR1 may be involved in the process by which PRP promotes the osteogenic differentiation of hADSCs. In the present study, total RNA samples from the OM and PRP groups were sequenced by high-throughput sequencing on day 14, and the differential miRNA and mRNA expression profiles were obtained to identify the miRNAs and genes involved in PRP-induced osteogenic differentiation of hADSCs.

ADSCs have the advantages of a high proliferation rate and antifibrotic, antiapoptotic, anti-inflammatory, and immunoregulatory effects [22], and they have the ability to differentiate into multiple different cell types. Through paracrine mechanisms, ADSCs have great potential in wound healing [23], treatment of cardiovascular diseases [24], nerve regeneration [25], cartilage repair [26], and other fields. Many cell experiments and animal studies have shown that in a specific induction environment, ADSCs can achieve osteogenic differentiation or form bone tissue in vivo, thereby providing a new approach for the clinical treatment of alveolar bone defects. Improving the osteogenic differentiation ability of ADSCs is a research hotspot. Coculture with other cells, the addition of osteogenic inducible factors and the modification of ADSCs are all effective ways to promote the osteogenic differentiation of ADSCs. Studies have shown that coculture of ADSCs and umbilical vein endothelial cells improves the proliferation, osteogenesis, and angiogenesis of ADSCs [27]. Nel-like protein 1 (NELL1) induces osteogenic differentiation of ADSCs in vitro and promotes the expression of osteogenic genes, such as ALP, COL1A1, OCN, and Runx2. The combined application of NELL1 and ADSCs improves bone microstructure, significantly increases the bone volume fraction, significantly increases the number of bone trabeculae, forms new bone, and effectively corrects severe bone loss in osteogenic imperfection mouse models [28]. circRNA-vGLL3 positively regulates the osteogenic differentiation of ADSCs, and circRNA-vGLL3-modified ADSCs significantly promote the repair of cranial defects of critical size in rats and increase new bone formation [29].

PRP was first reported for cardiac surgery in the late 1980s and later used for treatment in orthopaedic surgery, gynaecology, urology, sports injuries, and osteoarthritis [30–33]. PRP is derived from autologous blood in a minimally invasive procedure, avoids immune rejection, and has the advantages of being easy to obtain and simple to prepare. Platelets, as the main component of PRP, have a concentration 3-5 times that in whole blood, contain more than 1,100 different proteins and produce more than 1,500 bioactive factors [34]. PRP plays an important role in cell proliferation, migration, and differentiation, and it promotes wound healing and repairs bone defects.

Different preclinical and clinical studies have confirmed the biosafety of ADSCs [35], and it may only be a matter of time before ADSCs are widely used in the treatment of alveolar bone defects. The osteogenesis regulation mechanism of ADSCs is complex and involves many genes. Drawing a complete gene regulation network map and further studying the molecular mechanism are helpful to promote the clinical transformation of ADSCs. At present, there has been no research on the mechanism by which PRP promotes the osteogenesis of ADSCs. In the present study, miRNA sequencing and mRNA sequencing were performed on total RNA samples from the OM and PRP groups using high-throughput sequencing technology, aiming to explore the gene regulation mechanism by which PRP promotes the osteogenesis of ADSCs.

High-throughput sequencing technology can be used for in-depth analysis of the genome of species and provides an effective technical means for the discovery of miRNAs and the mining of miRNA biological regulatory pathways. Through miRNA sequencing and mRNA sequencing, 82 differentially expressed miRNAs and 1146 differentially expressed mRNAs were obtained in the present study. We performed GO enrichment analysis, KEGG pathway enrichment analysis, selection of osteogenic GO terms/pathways, and miRNA/mRNA combined analysis. Finally, 28 miRNA/mRNA reverse regulatory relationships that may be associated with osteogenesis were obtained (Table 4). In the present study, the following four relationships were selected for qRT–PCR verification: (1) downregulation of hsa-miR-212-5p/upregulation of CNR1, (2) downregulation of hsa-miR-495-3p_R+1/upregulation of CNR1, (3) upregulation of hsa-miR-204-3p/downregulation of LEP, and (4) upregulation of hsa-miR-204-3p/downregulation of GREM1. The results showed that the expression level of hsa-miR-204-3p was significantly downregulated (*P* < 0.05), which was the opposite of the sequencing results. However, we could not verify whether hsa-miR-204-3p upregulation/LEP downregulation and hsa-miR-204-3p upregulation/Grem1 downregulation are involved in the osteogenic differentiation of hADSCs.

The human bone morphogenetic protein antagonist, GREM1, was the focus of this study. GREM1 belongs to the DNA family of secretory BMP antagonists [36] and plays an important role in kidney and bone development [37, 38]. Grem1-MUT mice develop severe limb bone deformities [39]. GREM1 inhibits the activity and osteogenic differentiation of human BMSCs, and inhibition of the GREM1 expression improves cell viability and osteogenic differentiation induced by BMP-2 [40]. The specific overexpression of Grem1 in mouse bone tissue leads to severe symptoms of osteoporosis. The removal of GREM1 in bone tissue increases bone formation and trabecular volume [41]. Liu et al. showed that the overexpression of GREM1 in ADSCs reduces the activity of alkaline phosphatase and inhibits the expression of Runx2, OCN, and other osteogenic genes. Knockout of Grem1 in ADSCs enhances alkaline phosphatase activity and promotes the expression of osteogenic genes. Therefore, these findings suggest that GREM1 inhibits the osteogenic differentiation of ADSCs [36]. The above results are consistent with the conclusion of this study; that is, the reduced expression of GREM1 is conducive to osteogenic differentiation and bone formation of stem cells. According to the regulatory relationship in Table 4, GREM1 may be negatively regulated by hsa-miR-204-3p and play a role in the osteogenic differentiation of hADSCs, which will be our future research direction, aiming to lay a foundation for the preclinical study of GREM1 combined with hADSCs in the treatment of alveolar bone defects.

The qRT–PCR verification results of hsa-miR-212-5p, hsa-miR-495-3p_r+1, and CNR1 were consistent with the sequencing results; that is, hsa-miR-212-5p was downregulated, and CNR1 was upregulated (*P* < 0.05). The results of miRNA/mRNA combined analysis and dual-luciferase assays indicated that the downregulation of hsa-miR-212-5p and the upregulation of CNR1 are involved in the process by which PRP promotes the osteogenic differentiation of hADSCs. miR-212-5p plays an important role in the occurrence, development, treatment, and prognosis of renal cancer [42], lung cancer [43], breast cancer [44], rectal cancer [45], and aneurysms [46]. To date, however, there has been no report on the role of miR-212-5p in osteogenesis. The endocannabinoid system plays an important role in physiological processes, such as appetite control, energy balance, pain perception, and immune response [47]. Several studies have shown that the endocannabinoid system is involved in bone metabolism [48, 49]. Human osteoclasts also express CNR1 and type 2 cannabinoid receptor (CNR2) [50], and the regulation of CNR1 in the endocannabinoid system may be an important therapeutic tool for human bone diseases. CNR1 is necessary for the survival of bone marrow mesenchymal stem cells and is upregulated during osteogenic differentiation [51]. Idris et al. showed that CNR1 drug blockade stimulates the differentiation of adipocytes and inhibits the differentiation of bone cells, and they reported that age-related osteoporosis occurs in CNR1-deficient mice [52]. Other studies have shown that CNR1 signaling positively regulates bone growth through upregulation of bone formation and downregulation of bone absorption, and CNR1-deficient mice show a low bone mass phenotype with reduced trabecular density and bone volume fraction [53]. Together, these studies confirm the important role of CNR1 in bone formation, which is consistent with the conclusion of the present study, namely, the increased expression of CNR1 is conducive to the osteogenic differentiation and bone formation abilities of stem cells.

In conclusion, the present study demonstrated that PRP is noncytotoxic and promotes the osteogenic differentiation of hADSCs by downregulating hsa-miR-212-5p and upregulating CNR1. The differentially expressed miRNA profiles and mRNA profiles of PRP promoting the osteogenic differentiation of hADSCs were identified listed, and the targeting relationship between hsa-miR-212-5p and CNR1 was verified. The present study explored the mechanism by which PRP promotes the osteogenic differentiation of hADSCs, thereby contributing to the improvement of the gene network map of hADSC osteogenic differentiation, providing a reference for related studies and laying a preliminary foundation for the clinical application of hADSCs in the treatment of alveolar bone defects.

Stem cells play an increasingly important role in regenerative medicine. PRP regulates the proliferation and differentiation of stem cells. The combination of hADSCs and PRP is an attractive approach for periodontal tissue regeneration, but research in this area is still in its infancy [54, 55]. Although collection and treatment techniques for ADSCs have been standardized and clinical applications are being reported [56], the mechanisms are not fully understood. Due to the difference in material form and preparation technology, the published results for PRP are often contradictory [57], and a consensus has not been reached for the optimal PRP purification protocol [58], which will be the focus of our future research. In addition, PRP regulates the key growth factors of stem cell proliferation and differentiation, and the signaling pathways involved will be studied. The benefits and risks in the field of stem cell regeneration need to be fully studied and validated in a large number of patients before they can be clinically utilized.

## 5. Conclusion

PRP promotes the osteogenic differentiation of hADSCs, and the downregulation of hsa-miR-212-5p and the upregulation of CNR1 may be involved in this process. hsa-miR-212-5p binds to the 3′ UTR-specific site of CNR1.

## Figures and Tables

**Figure 1:** Characterization and identification of hADSCs. (a) Third-generation hADSCs (×40 magnification). (b) Third-generation hADSCs (×100 magnification). (c) Immunophenotypical analysis of hADSCs by flow cytometry. hADSCs were positive for CD73, CD90, and CD105 but negative for CD34 and CD45. (d) Alizarin Red staining showing calcium nodules (stained red). (e) Oil Red O staining showing lipid droplets (stained red). (f) Alcian blue staining showing the internal acid mucopolysaccharide in cartilage tissue (stained blue).

**Figure 2:** PRP promotes the proliferation of hADSCs and the formation of calcium nodules. (a) No calcium nodules were formed in the CON group as indicated by the lack of Alizarin Red staining. (b) Few calcium nodules were formed in the OM group as indicated by Alizarin Red staining. (c) Many calcium nodules were formed in the PRP group as indicated by Alizarin Red staining. (d) The effect of the different culture media on the proliferation of hADSCs was evaluated by a CCK-8 assay (^∗^ vs. con, *P* < 0.05, *n* = 5). (e) Change in the expression of Runx2 (^∗^ vs. OM, *P* < 0.05, *n* = 3).

**Figure 3:** Results of miRNA sequencing and mRNA sequencing. (a) Heat map of differentially expressed miRNAs. (b) Histogram for the GO enrichment analysis of differentially expressed miRNA target genes. (c) Volcano map of differentially expressed genes (*P* > 0.05). (d) Histogram of GO enrichment analysis results for 156 osteogenesis-related genes. (e) Scatter plot of KEGG enrichment analysis results for 102 osteogenesis-related genes. In the scatter diagram, the size of the dot represents the number of differentially expressed genes, and the color of the dot represents the *P* value of the enrichment analysis. *P* < 0.05 indicates significant enrichment. (f) Analysis of miRNA and mRNA sequencing results and flow chart of miRNA/mRNA combined analysis.

**Figure 4:** The relative expression levels of hsa-miR-204-3p, hsa-miR-212-5p, hsa-miR-495-3p_r+1, LEP, GREM1, and CNR1 were verified by qRT–PCR (^∗^ vs. OM, *P* < 0.05, *n* = 3).

**Figure 5:** The downregulation of hsa-miR-212-5p and the upregulation of CNR1 may be involved during the PRP-mediated osteogenic differentiation process. (a) Relative mRNA expression levels of ALP, Runx2, OCN, COL1A1, CNR1, and has-miR-212-5p. (b) Western blot analysis of ALP, Runx2, OCN, COL1A1, and CNR1 protein expression levels. *β*-Actin was used as an internal control (^∗^ vs. OM, *P* < 0.05, *n* = 3). (c) Predicted binding site of hsa-miR-212-5p in the 3′ UTR of CNR1 mRNA. (d) The hsa-miR-212-5p overexpression inhibited the luciferase activity of WT-CNR1 cells compared to NC cells, whereas the luciferase activity of MUT cells was not significantly altered by the hsa-miR-212-5p overexpression. WT: wild-type; MUT: mutant; NC: negative control (^∗^ vs. NC, *P* < 0.05, *n* = 3).

**Table 1:** Sequences of primers used in this study.

Gene	Forward primer (5′-3′)	Reversed primer (5′-3′)
CNR1	CCTGGTGCTGTGCGTCAT	CGTTGCGGCTATCTTTGC
GREM1	ATCATCAACCGCTTCTGT	GAGCAGGACTGAAAGGAA
LEP	TTGTCACCAGGATCAATGA	CATCTTGGATAAGGTCAGGA
hsa-miR-212-5p	GTGACGGCTTACTGTCGTATCCA	GTCGTATCCAGTGCAGGGTCCGAGGTATTCGCACTGGATACGACAGTAAGCAGTCTAGAGCCAAGGT
hsa-miR-204-3p	CGTGGGAAGGCAAAGGGAC	GTCGTATCCAGTGCAGGGTCCGAGGTATTCGCACTGGATACGACACGTCCCTTTGCCTTCCCAGC
hsa-miR-495-3p_R+1	GGAGAGGCACTTCTTTGTCGTAT	GTCGTATCCAGTGCAGGGTCCGAGGTATTCGCACTGGATACGACAAAGAAGTGCACCATGTTTGTTT
COL1A1	CGAAGACATCCCACCAATC	ATCACGTCATCGCACAACA
ALP	TTGGGCTGTGGAAGGCTCTG	TTCCTCCTTGTTGGGTTTGG
Runx2	TCAGGCATGTCCCTCGGTAT	GGCTTCCATCAGCGTCAA
OCN	GAAGAGGAGGGAGAATGTTG	CACTGAAGGGTCTGGTAGGA
GAPDH	TGCACCACCAACTGCTTAGC	GGCATGGACTGTGGTCATGAG

**Table 2:** Differential miRNA expression profile.

miRNA	FC (PRP/OM)	log2 (FC)	*P* value	Regulation
hsa-miR-370-3p	2.09	1.06	0.0018	Down
hsa-miR-1248_R-4	0.49	-1.01	0.0026	Up
hsa-miR-212-5p	3.39	1.76	0.0045	Down
hsa-mir-7110-p3_1ss1TC	0.32	-1.64	0.0045	Up
hsa-miR-9901_L+3R-2	0.18	-2.47	0.0071	Up
hsa-miR-496_L-2R+1	2.21	1.14	0.0075	Down
hsa-miR-5684_L-1R-1_1ss6TC	0.11	-3.16	0.0080	Up
ssc-mir-1285-p3_1ss20TA	0.49	-1.04	0.0089	Up
hsa-miR-4521_R+3	0.30	-1.74	0.0092	Up
hsa-miR-126-3p	3.08	1.62	0.0097	Down
bta-mir-2904-2-p3	0.46	-1.14	0.0126	Up
mmu-mir-8112-p5_1ss13CT	0.34	-1.55	0.0139	Up
hsa-miR-31-3p_R+1	3.63	1.86	0.0162	Down
hsa-miR-337-3p	2.17	1.12	0.0164	Down
hsa-mir-9902-1-p3_1ss13GC	0.38	-1.40	0.0174	Up
hsa-miR-1260a_L+1_1ss10TG	0.46	-1.12	0.0195	Up
mmu-mir-6236-p5_3	0.47	-1.08	0.0200	Up
mmu-mir-6236-p5_2	0.47	-1.08	0.0200	Up
mmu-mir-6236-p5_1	0.47	-1.08	0.0200	Up
mmu-mir-6236-p5_4	0.47	-1.08	0.0200	Up
mmu-mir-6236-p3_4	0.47	-1.08	0.0200	Up
ssc-mir-4332-p5_1ss11CA	0.31	-1.68	0.0217	Up
Hha-miR-4521_R+3	2.55	1.35	0.0217	Down
mmu-mir-6240-p5_1ss12TG_1	0.47	-1.08	0.0280	Up
mmu-mir-6240-p5_1ss12TG_2	0.47	-1.08	0.0280	Up
ssc-mir-4332-p5_1ss12CA	0.32	-1.64	0.0298	Up
hsa-miR-5010-3p_R+1	2.15	1.11	0.0327	Down
bta-miR-2887_L-2R+5	0.33	-1.59	0.0328	Up
bta-mir-2887-1-p5_1ss24AT	0.31	-1.70	0.0350	Up
hsa-miR-4485-5p_L+2R+2	0.18	-2.51	0.0355	Up
hsa-miR-204-3p	0.15	-2.72	0.0370	Up
bta-miR-11987_L-1R-1_1ss8TA	0.43	-1.21	0.0374	Up
ssc-mir-1285-p5_1ss23TC	0.45	-1.16	0.0375	Up
hsa-miR-138-5p	0.21	-2.28	0.0407	Up
hsa-miR-495-3p_R+1	2.30	1.20	0.0429	Down
hsa-miR-146b-3p	2.40	1.26	0.0429	Down
eca-mir-8986a-p5_1ss1GA	0.48	-1.06	0.0430	Up
bta-mir-2887-1-p3_1ss18AT	0.35	-1.50	0.0439	Up
bta-miR-2887_R+2	0.32	-1.64	0.0439	Up
mdo-miR-152-3p_R+3	5.47	2.45	0.0440	Down
hsa-miR-148a-5p	2.92	1.55	0.0441	Down
hsa-miR-618	4.78	2.26	0.0473	Down
hsa-miR-542-5p_R-1	7.90	2.98	0.0497	Down

**Table 3:** Differential mRNA expression profile associated with PRP promoting osteogenic differentiation of hADSCs.

mRNA name	FC	log2 (FC)	*P* value	Regulation
FABP3	6.83	2.77	≤0.001	Down
TUBA1A	2.94	1.56	≤0.001	Down
MVD	2.90	1.53	≤0.001	Down
GPC3	2.71	1.44	≤0.001	Down
LEP	2.58	1.37	≤0.001	Down
GREM1	2.50	1.32	≤0.001	Down
CTHRC1	2.44	1.29	≤0.001	Down
LGALS1	2.11	1.07	≤0.001	Down
F2R	0.49	-1.02	≤0.001	Up
GRB2	0.47	-1.08	≤0.001	Up
SPTBN1	0.47	-1.08	≤0.001	Up
FOXO1	0.47	-1.09	≤0.001	Up
CDC42EP3	0.46	-1.11	≤0.001	Up
PLPP3	0.46	-1.12	≤0.001	Up
PTK2B	0.46	-1.13	≤0.001	Up
GTF3C5	0.43	-1.20	≤0.001	Up
DNAJA3	0.42	-1.25	≤0.001	Up
KAT2A	0.36	-1.47	≤0.001	Up
CNR1	0.27	-1.90	≤0.001	Up
ID1	0.22	-2.21	≤0.001	Up

**Table 4:** miRNA/mRNA osteogenic regulation relationships.

MicroRNA information				mRNA information			
miRNA	FC	Regulation	*P* value	mRNA	FC	Regulation	*P* value
hsa-miR-212-5p	3.39	Down	≤0.001	CNR1	0.14	Up	≤0.001
hsa-miR-495-3p_R+1	2.30	Down	0.04	CNR1	0.14	Up	≤0.001
mdo-miR-152-3p_R+3	5.47	Down	0.04	CNR1	0.14	Up	≤0.001
bta-miR-2887_R+2	0.32	Up	0.04	LEP	2.58	Down	0.02
bta-mir-2887-1-p5_1ss24AT	0.31	Up	0.03	LEP	2.58	Down	0.02
hsa-miR-138-5p	0.21	Up	0.04	MVD	5.48	Down	≤0.001
hsa-miR-138-5p	0.21	Up	0.04	LEP	2.58	Down	0.02
hsa-miR-204-3p	0.15	Up	0.04	LEP	2.58	Down	0.02
hsa-miR-204-3p	0.15	Up	0.04	GREM1	2.56	Down	0.02
hsa-miR-204-3p	0.15	Up	0.04	CDC42EP3	43.27	Down	≤0.001
hsa-miR-5684_L-1R-1_1ss6TC	0.11	Up	0.01	LEP	2.58	Down	0.02
hsa-miR-5684_L-1R-1_1ss6TC	0.11	Up	0.01	GREM1	2.56	Down	0.02
hsa-mir-7110-p3_1ss1TC	0.32	Up	0.00	GREM1	2.56	Down	0.02
hsa-miR-9901_L+3R-2	0.18	Up	0.01	FABP3	57.81	Down	≤0.001
hsa-miR-9901_L+3R-2	0.18	Up	0.01	FABP3	8.50	Down	≤0.001
hsa-mir-9902-1-p3_1ss13GC	0.38	Up	0.02	LEP	2.58	Down	0.02
hsa-mir-9902-1-p3_1ss13GC	0.38	Up	0.02	GREM1	2.56	Down	0.02
mmu-mir-6236-p3_4	0.47	Up	0.02	GREM1	2.56	Down	0.02
mmu-mir-6236-p3_4	0.47	Up	0.02	CDC42EP3	43.27	Down	≤0.001
mmu-mir-6236-p5_3	0.47	Up	0.02	GREM1	2.56	Down	0.02
mmu-mir-6236-p5_3	0.47	Up	0.02	CDC42EP3	43.27	Down	≤0.001
mmu-mir-6236-p5_4	0.47	Up	0.02	LEP	2.58	Down	0.02
mmu-mir-6236-p5_4	0.47	Up	0.02	CDC42EP3	43.27	Down	≤0.001
mmu-mir-6240-p5_1ss12TG_1	0.47	Up	0.03	GREM1	2.56	Down	0.02
mmu-mir-6240-p5_1ss12TG_2	0.47	Up	0.03	GREM1	2.56	Down	0.02
mmu-mir-8112-p5_1ss13CT	0.34	Up	0.01	CDC42EP3	43.27	Down	≤0.001
ssc-mir-4332-p5_1ss11CA	0.31	Up	0.02	GREM1	2.56	Down	0.02
ssc-mir-4332-p5_1ss12CA	0.32	Up	0.03	GREM1	2.56	Down	0.02

## Data Availability

The data used to support the findings of this study are available from the corresponding author upon request.

## References

[1] Coşkun İ., Kaya B. (2019). Appraisal of the relationship between tooth inclination, dehiscence, fenestration, and sagittal skeletal pattern with cone beam computed tomography. *The Angle Orthodontist*.

[2] Amit G., Jps K., Pankaj B., Suchinder S., Parul B. (2012). Periodontally accelerated osteogenic orthodontics (PAOO) - a review. *Journal of Clinical and Experimental Dentistry*.

[3] Kamal A. T., Malik D. E. S., Fida M., Sukhia R. H. (2019). DL'orthodontie acceleree par stimulation osteogenique du parodonte ameliore-t- elle les resultats du traitement orthodontique ? Revue systematique et meta- analyse. *International Orthodontics*.

[4] Fei D., Wang Y., Zhai Q. (2021). KAT6A regulates stemness of aging bone marrow-derived mesenchymal stem cells through Nrf2/ARE signaling pathway. *Stem Cell Research & Therapy*.

[5] Chen L., Zhang R. Y., Xie J. (2021). STAT3 activation by catalpol promotes osteogenesis-angiogenesis coupling, thus accelerating osteoporotic bone repair. *Stem Cell Research & Therapy*.

[6] Li Q., Yang G., Li J. (2020). Stem cell therapies for periodontal tissue regeneration: a network meta-analysis of preclinical studies. *Stem Cell Research & Therapy*.

[7] Tavakolinejad S., Khosravi M., Mashkani B. (2014). The effect of human platelet-rich plasma on adipose-derived stem cell proliferation and osteogenic differentiation. *Iranian Biomedical Journal*.

[8] Ding G., Liu Y., Wang W. (2010). Allogeneic periodontal ligament stem cell therapy for periodontitis in swine. *Stem Cells*.

[9] Liao D., Gong P., Li X., Tan Z., Yuan Q. (2010). Co-culture with Schwann cells is an effective way for adipose-derived stem cells neural transdifferentiation. *Archives of Medical Science*.

[10] Tsuji W., Rubin J. P., Marra K. G. (2014). Adipose-derived stem cells: implications in tissue regeneration. *World Journal of Stem Cells*.

[11] Le A. D., Enweze L., De Baun M. R., Dragoo J. L. (2018). Current clinical recommendations for use of platelet-rich plasma. *Current Reviews in Musculoskeletal Medicine*.

[12] Dragoo J. L., Braun H. J., Durham J. L. (2012). Comparison of the acute inflammatory response of two commercial platelet-rich plasma systems in healthy rabbit tendons. *The American Journal of Sports Medicine*.

[13] Tajima S., Tobita M., Orbay H., Hyakusoku H., Mizuno H. (2015). Direct and indirect effects of a combination of adipose-derived stem cells and platelet-rich plasma on bone regeneration. *Tissue Engineering. Part A*.

[14] Donadeu F. X., Sontakke S. D., Ioannidis J. (2016). MicroRNA indicators of follicular steroidogenesis. *Reproduction, Fertility, and Development*.

[15] Cai Y., Yu X., Hu S., Yu J. (2009). A brief review on the mechanisms of miRNA regulation. *Genomics, Proteomics & Bioinformatics*.

[16] Li S., Hu C., Li J. (2016). Effect of miR-26a-5p on the Wnt/Ca2+ pathway and osteogenic differentiation of mouse adipose-derived mesenchymal stem cells. *Calcified Tissue International*.

[17] Liu X., Zhu W., Wang L., Wu J., Ding F., Song Y. (2019). miR-145-5p suppresses osteogenic differentiation of adipose-derived stem cells by targeting semaphorin 3A. *In Vitro Cellular & Developmental Biology. Animal*.

[18] Yang X. M., Song Y. Q., Li L., Liu D. M., Chen G. D. (2021). miR-1249-5p regulates the osteogenic differentiation of ADSCs by targeting PDX1. *Journal of Orthopaedic Surgery and Research*.

[19] Xie Q., Wang Z., Zhou H. (2016). The role of miR-135-modified adipose-derived mesenchymal stem cells in bone regeneration. *Biomaterials*.

[20] Agarwal V., Bell G. W., Nam J. W., Bartel D. P. (2015). Predicting effective microRNA target sites in mammalian mRNAs. *eLife*.

[21] Betel D., Koppal A., Agius P., Sander C., Leslie C. (2010). Comprehensive modeling of microRNA targets predicts functional non-conserved and non-canonical sites. *Genome Biology*.

[22] Sheykhhasan M., Wong J. K. L., Seifalian A. M. (2019). Human adipose-derived stem cells with great therapeutic potential. *Current Stem Cell Research & Therapy*.

[23] Mazini L., Rochette L., Admou B., Amal S., Malka G. (2020). Hopes and limits of adipose-derived stem cells (ADSCs) and mesenchymal stem cells (MSCs) in Wound Healing. *International Journal of Molecular Sciences*.

[24] Huang H., Xu Z., Qi Y. (2020). Exosomes from *SIRT1* -overexpressing ADSCs restore cardiac function by improving angiogenic function of EPCs. *Molecular Therapy--Nucleic Acids*.

[25] Zheng Z., Liu J. (2019). GDNF-ADSCs-APG embedding enhances sciatic nerve regeneration after electrical injury in a rat model. *Journal of Cellular Biochemistry*.

[26] Li X., Wang M., Jing X. (2018). Bone marrow- and adipose tissue-derived mesenchymal stem cells: characterization, differentiation, and applications in cartilage tissue engineering. *Critical Reviews in Eukaryotic Gene Expression*.

[27] Mutschall H., Winkler S., Weisbach V., Arkudas A., Horch R. E., Steiner D. (2020). Bone tissue engineering using adipose-derived stem cells and endothelial cells: effects of the cell ratio. *Journal of Cellular and Molecular Medicine*.

[28] Liu Y., Ju M., Wang Z. (2020). The synergistic effect of NELL1 and adipose-derived stem cells on promoting bone formation in osteogenesis imperfecta treatment. *Biomedicine & Pharmacotherapy*.

[29] Zhang D., Ni N., Wang Y. (2021). CircRNA-vgll3 promotes osteogenic differentiation of adipose-derived mesenchymal stem cells via modulating miRNA-dependent integrin *α*5 expression. *Cell Death and Differentiation*.

[30] Gupta S., Paliczak A., Delgado D. (2021). Evidence-based indications of platelet-rich plasma therapy. *Expert Review of Hematology*.

[31] Belk J. W., Kraeutler M. J., Houck D. A., Goodrich J. A., Dragoo J. L., McCarty E. C. (2021). Platelet-rich plasma versus hyaluronic acid for knee osteoarthritis: a systematic review and meta-analysis of randomized controlled trials. *The American Journal of Sports Medicine*.

[32] Medina-Porqueres I., Ortega-Castillo M., Muriel-Garcia A. (2021). Effectiveness of platelet-rich plasma in the management of hip osteoarthritis: a systematic review and meta-analysis. *Clinical Rheumatology*.

[33] Altamura S. A., Di Martino A., Andriolo L. (2020). Platelet-rich plasma for sport-active patients with knee osteoarthritis: limited return to sport. *BioMed Research International*.

[34] Boswell S. G., Cole B. J., Sundman E. A., Karas V., Fortier L. A. (2012). Platelet-rich plasma: a milieu of bioactive factors. *Arthroscopy*.

[35] Qomi R. T., Sheykhhasan M. (2017). Adipose-derived stromal cell in regenerative medicine: a review. *World Journal of Stem Cells*.

[36] Liu H., Han X., Yang H. (2021). GREM1 inhibits osteogenic differentiation, senescence and BMP transcription of adipose-derived stem cells. *Connective Tissue Research*.

[37] Tatsinkam A. J., Rune N., Smith J., Norman J. T., Mulloy B., Rider C. C. (2017). The binding of the bone morphogenetic protein antagonist gremlin to kidney heparan sulfate: such binding is not essential for BMP antagonism. *The International Iournal of Biochemistry & Cell Biology*.

[38] Huang X., Post J. N., Zhong L. (2018). Dickkopf-related protein 1 and gremlin 1 show different response than frizzled-related protein in human synovial fluid following knee injury and in patients with osteoarthritis. *Osteoarthritis and Cartilage*.

[39] Canalis E., Parker K., Zanotti S. (2012). Gremlin1 is required for skeletal development and postnatal skeletal homeostasis. *Journal of Cellular Physiology*.

[40] Hu K., Sun H., Gui B., Sui C. (2017). Gremlin-1 suppression increases BMP-2-induced osteogenesis of human mesenchymal stem cells. *Molecular Medicine Reports*.

[41] Gazzerro E., Smerdel-Ramoya A., Zanotti S. (2007). Conditional deletion of gremlin causes a transient increase in bone formation and none mass. *The Journal of Biological Chemistry*.

[42] Deng J. H., Zheng G. Y., Li H. Z., Ji Z. G. (2019). MiR-212-5p inhibits the malignant behavior of clear cell renal cell carcinoma cells by targeting TBX15. *European Review for Medical and Pharmacological Sciences*.

[43] Chen F. F., Sun N., Wang Y. (2020). miR-212-5p exerts tumor promoter function by regulating the Id3/PI3K/Akt axis in lung adenocarcinoma cells. *Journal of Cellular Physiology*.

[44] Lv Z. D., Yang D. X., Liu X. P. (2018). miR-212-5p suppresses the epithelial-mesenchymal transition in triple-negative breast cancer by targeting Prrx2. *Cellular Physiology and Biochemistry*.

[45] Du F., Li Z., Zhang G. (2020). SIRT2, a direct target of miR-212-5p, suppresses the proliferation and metastasis of colorectal cancer cells. *Journal of Cellular and Molecular Medicine*.

[46] Tian Z., Sun Y., Sun X., Wang J., Jiang T. (2020). LINC00473 inhibits vascular smooth muscle cell viability to promote aneurysm formation via miR-212-5p/BASP1 axis. *European Journal of Pharmacology*.

[47] Khalid A. B., Goodyear S. R., Ross R. A., Aspden R. M. (2016). Mechanical and material properties of cortical and trabecular bone from cannabinoid receptor-1-null (*Cnr1*^−/−^) mice. *Medical Engineering & Physics*.

[48] Sophocleous A., Marino S., Kabir D., Ralston S. H., Idris A. I. (2017). Combined deficiency of the Cnr1 and Cnr2 receptors protects against age-related bone loss by osteoclast inhibition. *Aging Cell*.

[49] Zhang C., Ma J., Chen G., Fu D., Li L., Li M. (2015). Evaluation of common variants in CNR2 gene for bone mineral density and osteoporosis susceptibility in postmenopausal women of Han Chinese. *Osteoporosis International*.

[50] Whyte L. S., Ford L., Ridge S. A., Cameron G. A., Rogers M. J., Ross R. A. (2012). Cannabinoids and bone: endocannabinoids modulate human osteoclast function in vitro. *British Journal of Pharmacology*.

[51] Gowran A., McKayed K., Campbell V. A. (2013). The cannabinoid receptor type 1 is essential for mesenchymal stem cell survival and differentiation: implications for bone health. *Stem Cells International*.

[52] Idris A. I., Sophocleous A., Landao-Bassonga E. (2009). Cannabinoid receptor type 1 protects against age- related osteoporosis by regulating osteoblast and adipocyte differentiation in marrow stromal cells. *Cell Metabolism*.

[53] Tam J., Ofek O., Fride E. (2006). Involvement of neuronal cannabinoid receptor CB1 in regulation of bone mass and bone remodeling. *Molecular Pharmacology*.

[54] Tobita M., Morikuni H. (2013). Adipose-derived stem cells and platelet-rich plasma: the keys to functional periodontal tissue engineering. *Current Stem Cell Research & Therapy*.

[55] James I. B., Coleman S. R., Rubin J. P. (2016). Fat, stem cells, and platelet-rich plasma. *Clinics in Plastic Surgery*.

[56] Gentile P., Orlandi A., Scioli M. G., di Pasquali C., Bocchini I., Cervelli V. (2012). Concise review: adipose-derived stromal vascular fraction cells and platelet-rich plasma: basic and clinical implications for tissue engineering therapies in regenerative surgery. *Stem Cells Translational Medicine*.

[57] Gentile P., Scioli M. G., Bielli A., Orlandi A., Cervelli V. (2017). Concise review: the use of adipose-derived stromal vascular fraction cells and platelet rich plasma in regenerative plastic surgery. *Stem Cells*.

[58] Qian Y., Han Q., Chen W. (2017). Platelet-rich plasma derived growth factors contribute to stem cell differentiation in musculoskeletal regeneration. *Frontiers in Chemistry*.

